# Online Diagnosis and Classification of CT Images Collected by Internet of Things Using Deep Learning

**DOI:** 10.1155/2022/5373624

**Published:** 2022-03-19

**Authors:** Qiufang Ma

**Affiliations:** College of Big Data, Qingdao Huanghai University, Qingdao, Shandong 266427, China

## Abstract

Deep learning technology has recently played an important role in image, language processing, and feature extraction. In the past disease diagnosis, most medical staff fixed the images together for observation and then combined with their own work experience to judge. The diagnosis results are subjective, time-consuming, and inefficient. In order to improve the efficiency of diagnosis, this paper applies the deep learning algorithm to the online diagnosis and classification of CT images. Based on this, in this paper, the deep learning algorithm is applied to CT image online diagnosis and classification. Based on a brief analysis of the current situation of CT image classification, this paper proposes to use the Internet of things technology to collect CT image information and establishes the Internet of things to collect the CT image model. In view of image classification and diagnosis, the convolution neural network algorithm in the deep learning algorithm is proposed to diagnose and classify CT images, and several factors affecting the accuracy of classification are proposed, including the convolution number and network layer number. Using the CT image of the hospital brain for simulation analysis, the simulation results confirm the effectiveness of the deep learning algorithm. With the increase of convolution and network layer and the decrease of compensation, the accuracy of image classification will decline. Using the maximum pool method, reducing the step size can improve the classification effect. Using relu function as the activation function can improve the classification accuracy. In the process of large data set processing, appropriately adding a network layer can improve classification accuracy. In the diagnosis and analysis of brain CT images, the overall classification accuracy is close to 70%, and in the diagnosis of tumor diseases, the accuracy is higher, up to 80%.

## 1. Introduction

With the improvement of people's life quality, people's attention to health is also increasing. The development of medical equipment and technology provides support for the diagnosis and treatment of various diseases [1–5]. At present, there is much diagnostic equipment in the hospital, such as ultrasonic imaging technology, computed tomography, and positron emission tomography. Different equipment images have their own advantages and disadvantages. Among them, CT image is a common technology for disease diagnosis at present. This technology takes X-rays from different angles to form three-dimensional images and then synthesizes cross-sectional images, which has high application value in tumor diagnosis [6–9]. In the previous disease diagnosis, most of the medical staff fixed the images together for observation and then combined with their own work experience to judge; the diagnosis results are subjective, time-consuming, and inefficient [10, 11]. In image classification and diagnosis, computer-aided diagnosis technology has become a hot topic. CAD assisted in time can provide a lot of help for doctors to extract image feature information, can effectively reduce the workload of doctors, and also has important value in the early development of diseases [12–14]. In the process of massive data processing, it is generally considered that the model is complex enough to extract more information. With the development of artificial intelligence technology, in-depth learning technology has also been applied to image segmentation and processing [15–18]. The deep learning algorithm is a kind of machine learning algorithm, which is mainly used to solve problems that cannot be solved by shallow learning. At present, this algorithm has formed different types and plays an important role in image classification [19]. Based on this, in the research and analysis of this paper, we intend to use the Internet of things technology to collect CT images, take brain CT images as an example, use the deep learning algorithm to classify brain CT images, and realize image classification and disease diagnosis.

The researchers trained a 3D convolutional neural network (CNN) to analyze head CT images and determine if they contain acute nervous system diseases or noncritical findings. Although not as accurate as radiologists, it is found that the algorithm is much faster in providing notification of key findings in a simulated clinical environment. It is also effective to prioritize emergency cases in the simulated radiologist's work list. The deep learning project is the initial research, which launched the Mount Sinai Artificial Intelligence Research Alliance (aisinai), a group of health system scientists, doctors, and researchers, which is committed to developing medical AI to improve patient care and accurately help doctors diagnose diseases, according to researchers. In the future, researchers plan to compare and study the effects of weak and strong supervised classifiers and radiography and explore the best method to combine the two methods.

Based on the brief analysis of the current situation of CT image classification, this paper proposes to use the Internet of things technology to collect CT image information and establishes the CT image model of the Internet of things. The innovative contributions of this paper include the following: (1) For image classification and diagnosis, a convolution neural network algorithm based on deep learning is proposed to diagnose and classify CT images, and several factors affecting the classification accuracy are proposed. (2) The hospital brain CT images are used for simulation analysis, and the simulation results verify the effectiveness of the deep learning algorithm. (3) Using relu function as the activation function can improve the classification accuracy. In the process of large data set processing, appropriately adding a network layer can improve classification accuracy.

## 2. Related Word

Medical image is of great value to the diagnosis and treatment of diseases. Image classification can get disease performance types from massive data, and classification of a certain part can also provide an important role in disease prediction [20]. At present, computer-aided technology has been applied in medical image classification, and semiautomatic and full-automatic classification and diagnosis methods are the key topics of medical research [21]. Many scholars have studied medical image classification. In medical image classification, Lumini et al. used different preprocessing methods to construct an *n*-layer image, from which multilayer descriptors were extracted as feature vectors for support vector machine training. They thought that multilayer and texture descriptors could be combined to be superior to the standard single-layer method [22]. Dai et al. used the modal classification database of image clef competitions in 2011, 2012, and 2013; used the local binary pattern, color, and edge directionality descriptors, fuzzy color and texture histogram, and scale invariant feature transformation (and its variant opposite) as visual features, combined with TF-IDF weighted standard word package text representation; and added text features. The prediction performance is further improved [23]. Basabain proposed improvements for the image classification algorithm and designed a medical image classification algorithm based on the plsa-sow model [24]. Wu et al. have also proposed the *t*-harris texture corner extraction method, combined with the inherent characteristics of medical images, using the texture corner to establish the KAP digraph model [25]. Garali et al. also improved the image classification algorithm and proposed a new computer-aided diagnosis technology of AD brain PET image classification. The brain image was divided into 116 regions of interest (ROI) by using atlas, and some statistical features (mean, standard deviation, skewness, kurtosis, and entropy) on the histogram were calculated. The selected regions were sorted according to SPF and input to the support direction. In the SVM classifier, the result is the same or better than that of the whole brain voxel or 116 regions [26]. In the past, most of the algorithms were used to classify individual images, but few of them were used. In the research and analysis of this paper, the Internet of things was used to collect images, and the deep learning algorithm was used to diagnose and classify images.

## 3. Model Design

### 3.1. CT Image Acquisition Model

The Internet of things is to collect and analyze information by means of sensing and transmission, which improves the efficiency of information processing. At present, the Internet of things system covers the information sensing layer, data transmission layer, and processing layer, in which information sensing generally uses RFID technology to perceive things and realizes data transmission and processing through the Internet. At present, the Internet of things technology has a more mature technology, among which RFID technology is mostly used for image acquisition. This paper also uses this technology in CT image acquisition.

At present, in order to improve work efficiency, hospitals have begun to use algorithm systems to realize management, but image information acquisition technology has not been greatly improved. The emergence of RFID technology provides more convenience for image acquisition. RFID technology uses tags to identify images. When the performance enters the identification unit, it will be activated, and then, the information will be transmitted through the RF module. In combination with the image management methods currently adopted by the hospital, the Internet of things technology is used to achieve image acquisition. As shown in Figure 1, different kinds of image information are transmitted to his system through LAN, and then, the information is viewed through the system.

### 3.2. Deep Learning

Deep learning includes neural networks and deep learning. The artificial neural network is a model developed with computer technology [27, 28]. Since the model of artificial neural network appeared in the 1940s, it mathematicized biological neurons, regarded each processing unit as a node artificial neural network was inspired by biology, and based on the neural network abstracted rough candidate information from the perspective of information processing; the human neural network showed the characteristics of high fault tolerance and self-study in the past applications and was able to process and store signals and intelligently complete nonlinear problems. Assuming that there are *k* processing units, *X* information carried by processing units, and *W* connection weight, the output information of each unit can be expressed as follows:

(1) $$\begin{array}{c} y=f\left(\overset{k-1}{\underset{k=0}{\sum }}w_{k}x_{k}-\theta \right). \end{array}$$

In the formula, *f* represents the activation function, and the artificial neural network simulates the excitation and inhibition of neurons, with different output values. The artificial neural network model solves the nonlinear problem. After the weighted sum calculation, the results are input into the activation function to solve the nonlinear problem. Neural networks simulate the brain from knowledge acquisition and storage.

Deep learning can also be called hierarchical learning, which is a series of structural models. This algorithm is based on the artificial neural network and is also a part of the machine learning algorithm, with the emphasis on simulating human brain layer cells [29]. Deep learning solves high-level abstract problems by using multilevel nonlinear processing units. As long as these characteristics are satisfied, it can be called a deep learning model. There are many kinds of deep learning structures, most of which are based on the original structure and have their own application scope and conditions. The deep learning network contains at least one hidden layer. The multilayer structure model is more abstract, and its deep structure is used to describe the high-order characteristics of data. Many deep layer networks can generate samples from the network. The regional depth structure provides a description of data distribution, such as convolutional neural networks. The convolution neural network provides a learning model. Parameters can be calculated by the backpropagation algorithm. The trained neural network is applied to image information extraction. According to the similarity of images, the convolutional neural network can reduce the feature resolution, reduce the training parameters, and improve memory utilization. In the convolution neural network, convolution and pooling are special operations. These two operations can reduce dimensions, achieve the effect of reducing parameters, and improve training efficiency. Convolution includes continuous convolution and discrete convolution. The convolution neural network adopts discrete convolution, which is calculated by filters. The formula is expressed as follows:

(2) $$\begin{array}{c} X_{j}^{l}=f\left(\underset{i\in M_{f}}{\sum }X_{i}^{l-1}*k_{ij}^{l}+b_{j}^{l}\right), \end{array}$$

where *X* is the characteristic graph, *K* is the kernel function, and *F* is the activation function. Some of the properties of the image are consistent with other parts and have particularity, so the information obtained in the image can be applied to other parts. Convolution kernels generally contain three important features: size, number, and step size. The size of the convolution integral determines the number of feature graphs. It is generally believed that the more the number, the more the feature map. But it will also cause the increase of calculation parameters and complexity, so many experiments are needed.

For an image, there are certain similarities between adjacent or close pixel points. These similar pixel points can be simulated by one pixel point [30]. The pooling methods include the mean algorithm, maximum pooling method, and random pooling method. The mean pooling method selects the mean value from the adjacent eigenvalues, retains the image background information, and reduces the influence of the neighborhood on it. The maximum pooling method is to select the maximum value, retain more image texture information, and reduce the offset caused by parameter error. The random pooling method is to randomly select the maximum value in the adjacent area, and the larger the eigenvalue is, the easier it is to be selected.

In the deep learning algorithm, the convolutional neural network is a very representative method; this method combines the advantages of the detection algorithm, without reducing the speaking rate; the learning efficiency does not decline. This learning method also has high adaptability [31–33]. When a new learning sample is added, just remember to adjust the weight; it can improve the diagnosis rate. For example, in the diagnosis of diseases, image preprocessing can be done through regional growth, and the early samples can be saved in the database. The samples can be used to carry out error backpropagation and constantly adjust the parameters. When the error reaches a certain value, then use the sample data to test, and get the final diagnosis and classification results. In the convolution neural network, convolution processes the image, but this processing method belongs to the linear processing method. Many image data are not linearly distributed, so nonlinear processing is needed. The choice of activation function is very important for nonlinear processing. There are four kinds of activation functions commonly used. In this paper, relu function is used to simulate the process of brain neurons receiving signals being activated, which is more close to the reality of brain nerve activation. When the input value is less than 0, the output value is always 0. When the artificial neural network is trained, there may be less image data, so it needs to be processed to avoid overfitting. First, find more qualified data, increase the amount of data from the source, and increase the weight in each iteration to avoid overfitting.

In network training and learning, the effective improvement of machine learning promotes the development of the backpropagation algorithm. This paper also applies this algorithm in research and analysis. Suppose the data set has performance and there are *m* samples in the data set. For a single sample, the variance can be expressed as

(3) $$\begin{array}{c} J\left(W,b,x,y\right)=\frac{1}{2}{\left\|h_{w,b}\left(x\right)-y\right\|}^{2}. \end{array}$$

In the backpropagation algorithm, the smaller the value of the cost function, the better. Initialize the parameters *w* and *B*; the specific value cannot be exactly the same. Then, use the random gradient descent method to reduce the cost function. In the solution of partial derivative, backpropagation is very effective and can be expressed by residual. In the network parameter training, the output value of each layer can be obtained by forwarding to operation, and the difference with the ideal value is the residual value. In the application of the reverse algorithm, the connection weight is initialized first and assigned to a random value, and then, the output value is calculated by the conduction formula; the residual and partial derivative are calculated, and the weight is modified.

### 3.3. Model Structure Design

The structure of the neural network is determined by the connection between neurons; each neuron will be simulated. Taking neurons as network nodes, the model is constituted by power cases. In this traditional model, each input has its corresponding output value.

Caffe architecture provides a command line-oriented interface, which provides a possibility for the realization of the deep learning algorithm. Compared with other deep learning frameworks, this architecture method runs fast, has strong readability, is convenient for modification and improvement, and can be tested automatically. In the framework, net is used to represent the neural network model. Blob is the basic data structure of the framework. The dimension is from high to low. Blob provides a unified memory interface. When calculating, each layer of input and output needs buffer. The basic calculation unit of the framework is a layer, part of which has weight, and has two operation directions of backpropagation and forward propagation. The deep learning model includes three parameters: learning parameter, structure parameter, and training parameter. The learning parameters can be coefficients and weights. They are controlled according to the initialization parameters and generally do not interfere with the design manually. Once the structural parameters are set, they cannot be changed. The training parameters are used to control the convergence.

In order to better analyze the classification effect of deep learning neural networks, based on the alexnet architecture, select the activation function and network layer number, design different structure networks, and apply them to classification. Select multiple data sets, with each category containing tens of thousands of images, and take the image part as the training sample and the rest as the test sample. In the convolution layer, there are three important parameters. On the basis of the Caffe framework, a neural network is built to analyze the classification results under different convolutions and numbers. In Table 1, the training accuracy can reach more than 90%. With the increase of the number of convolution kernels, the classification error rate gradually decreases. Neurons connect with each other to form a complex model, and the performance is also related to the number. Because of the large amount of calculation, if a large network is constructed, the detection results may be affected. In this paper, a 7-layer convolution neural network is proposed. This model is automatically layered with supervision and outputs five tags. In the first part, we use a 13∗13 convolution kernel to extract the most typical features from CT images. With the increase of depth, feature extraction becomes more abstract.

In the pooling analysis, different pooling methods are selected for image classification. The results are shown in Table 2. From the data in the table, we can see that the maximum pooling method is more effective. When the window size is the same, with the reduction of the size, the classification accuracy will be improved. There are four kinds of activation functions commonly used; different functions have different deformations. In the analysis, these activation functions are analyzed, and then, the accuracy is measured in the classification task. Sigmoid function is applied to the shallow network. In the training network, you will cause data dispersion, and the effect is not very good. Tanh function has some improvement, but it will not solve the problem of gradient disappearance. The learning speed of the front hidden layer is lower than that of the back hidden layer. This phenomenon commonly exists in neural networks, which is called the vanishing gradient problem. For the solution, after pretraining, the whole network is fine-tuned. Hinton uses this method in training deep belief networks. After the pretraining of each layer is completed, he uses the BP algorithm to train the whole network. This idea is equivalent to looking for the local optimum first and then integrating it to find the global optimum. The emergence of relu function solves the problem of unilateral inhibition, and the accuracy measurement results also show that relu function is the best method to classify activation function.

Then, it analyzes the impact of network layers on the classification accuracy, analyzes the network structure, deletes a layer, with the layers having the same structure, and finds that there are some differences in the classification accuracy under different layers. The deeper the level, the richer the features, the better the classification effect. With the increase of layers, the parameter design also needs to be increased, and the number of network layers needs to be selected according to the actual situation.

## 4. Model Simulation Analysis

### 4.1. CT Image Data Preprocessing

In the simulation analysis, the data sets of hospitals are used to classify. These CT images are all from the hospital. The thickness of the layer when CT collects information is 3.75 mm. These images are all diagnosed and labeled by disease, and the boundary is very clear. The data set contains millions of image data, including 1.2 million training images, 50000 images to be verified, and 100000 images to be tested. Because of the great difference of different types of CT images, this paper takes human brain CT images as an example. The CT images are from the radiology department of the hospital, which are divided into five types, including normal brain image, brain tumor image, cerebral hemorrhage image, brain injury image, and cerebral infarction image.

CT image has the characteristics of high resolution, and all images will cover a large number of data. In order to ensure a higher learning effect, this paper uses MATLAB software to process CT images, process image resolution, and realize clutter removal. In this paper, based on the Caffe framework, all data need to be converted to the format before training, that is, LMDB format. This processing method can also improve the utilization of data through format.

In CT image diagnosis and classification, brain CT image is divided into five categories. In order to ensure the analysis effect, data sets are used to fit. The training set is selected randomly from the data set, and the images of some data sets are selected due to the limitation of conditions. After the training set is determined, a new training data folder and a verification data set are established. In addition, five folders corresponding to different image classifications are established, and the training images are collected in these folders. The CT images used in the experiment are all black-and-white images. In order to ensure the analysis effect, change the gray serial port to get the color image.

### 4.2. Experimental Result

In CT image analysis, a confusion matrix is used for classification and evaluation. This algorithm belongs to the visualization algorithm. Table 2 is a standard graph; row represents category value; list represents predicted value; TP represents true positive, that is to say, correct classification data; TN represents true negative, that is, correct classification health image; FP represents false positive; and FN represents false negative [34–41].

In the experimental analysis, first, use the accuracy to identify the image classification effect, then use the hit rate to view the classification effect, and judge the effectiveness of the algorithm. In the calculation, the accuracy rate represents the proportion of correct classification, and the hit rate refers to the percentage of correctly identified cases and model predicted cases.

In the convolution neural network model, leaky relu function is selected as the internal activation function, sigmoid function is selected as the outermost activation function, the maximum pooling method is adopted, the size is set to 2∗2, and the last full connection layer is fitted to improve the generalization ability. The volume integral network model is used to analyze medical images. The simulation analysis is completed in the Linux system. The weight of each layer is obtained by using the backpropagation algorithm and random gradient descent. 25 pictures are input in each iteration, and the weight learning rate is set to 0.01. When the number of iterations is more than 200, the weight is greatly reduced, and the paranoid learning rate is set to 0.02. After image preprocessing, transform format, generate mean value file, and add information to build the training model. Finally, the image data set is used to predict again to get the final model. Considering the small size of the image data set, the cross-validation method is used in training. The image is divided into 10 parts; then, the data is used to test, and finally, the average value of classification accuracy is obtained. According to the cross-validation method, the network model is obtained, and the figure is the result of the cross-validation. Using this model to classify medical CT images directly, the accuracy can reach 60% Figure 2.

The trained network model is used to analyze the image with high accuracy in detail. With the increase of the number of iterations, the value gradually decreases. In the test results, with the increase of the number of iterations, the accuracy is also stable. After more than 2500 times, there is little change. In the test process, the disease classification is analyzed by the confusion matrix of the network model, and Table 3 is the prediction result. The network model has a good effect on CT image classification diagnosis.

After determining the training set, you need to create a new training data folder and verify the data set. In CT image classification, the overall efficiency of the convolution neural network model established in this paper is more than 65%, and the hit rate of a single disease diagnosis is more than 80%, but the diagnostic effect of some diseases is relatively low, only 60%. In the application scene and image analysis, the deep learning algorithm is applied to the classification of brain CT images. At present, the diagnosis of brain CT images has been continuously studied. Subtle changes in the image may lead to some diseases, thus affecting the classification accuracy. In addition, the data set of brain CT images is small, which may lead to some errors.

## 5. Conclusion

At present, the deep learning algorithm has been paid more and more attention, and the technology is also improving. The application in medical CT images has also been paid more and more attention. In the research and analysis of this paper, the Internet of things technology is used to collect the CT image of the hospital, and the deep learning algorithm is used to detect and classify the image. Through experiments, the factors that affect the accuracy of convolution neural network classification are proposed. With the increase of convolution and network layers and the decrease of compensation, the accuracy of image classification will decline to some extent. Using the maximum pooling method, reducing the step size can improve the classification effect. Using relu function as activation function can improve the accuracy of classification. In the process of big data set processing, adding a network layer properly can improve the accuracy of classification. In the diagnosis and analysis of brain CT images, the overall classification accuracy is close to 70%, and in the diagnosis of tumor diseases, the accuracy is higher, reaching 80%. It needs to be pointed out that there are some defects in the research of this paper, which are limited by the experimental conditions. In the design of network models, the fitting environment is built. In the collection of CT images using the Internet of things, the article only designs a simple model, which is still in the trial stage. It also needs to improve the actual environment, build a more reasonable network model, and increase the size of the data set. The accuracy of classification can be improved by using CT images directly.

## Figures and Tables

**Figure 1:** CT image information acquisition.

**Figure 2:** Cross-validation results of CNN brainct network.

**Table 1:** Results of cifar-10 classification for networks with different convolution kernels.

First level convolution	Training accuracy	Test accuracy
18	90.6	83.2
12	91.3	82.6
24	91.5	84.5
36	92.3	86.7

**Table 2:** CT image information acquisition.

Confusion matrix		Predicted	
		Positive	Negative
Actual	Positive	TP	FP
	Negative	FN	TN

**Table 3:** Confusion matrix analysis results of network test.

Confusion matrix	Prediction results				
	Brain tumor	Cerebral infarction	Cerebral hemorrhage	Traumatic brain injury	Normal
Brain tumor	852	15	162	53	26
Cerebral infarction	0	526	0	11	452
Cerebral hemorrhage	126	25	715	163	12
Traumatic brain injury	135	6	228	638	1
Normal	11	316	18	15	648

## Data Availability

The data used to support the findings of this study are available from the corresponding author upon request.
